This article has been retracted.

# *Eucommia ulmoides* Oliver Extract, Aucubin, and Geniposide Enhance Lysosomal Activity to Regulate ER Stress and Hepatic Lipid Accumulation

**DOI:** 10.1371/journal.pone.0081349

**Published:** 2013-12-11

**Authors:** Hwa-Young Lee, Geum-Hwa Lee, Mi-Rin Lee, Hye-Kyung Kim, Nan-young Kim, Seung-Hyun Kim, Yong-Chul Lee, Hyung-Ryong Kim, Han-Jung Chae

**Affiliations:** 1 Department of Pharmacology and Institute of Cardiovascular Research, Medical School, Chonbuk National University, Jeonju, Chonbuk, Republic of Korea; 2 College of Pharmacy, Yonsei Institute of Pharmaceutical Sciences, Yonsei University, Incheon, Korea, Republic of Korea; 3 Department of Internal Medicine, Chonbuk National University Medical School, Jeonju, Korea; 4 Department of Dental Pharmacology, School of Dentistry, Wonkwang University, Iksan, Chonbuk, Republic of Korea; University of Catania, Italy

## Abstract

*Eucommia ulmoides* Oliver is a natural product widely used as a dietary supplement and medicinal plant. Here, we examined the potential regulatory effects of *Eucommia ulmoides* Oliver extracts (EUE) on hepatic dyslipidemia and its related mechanisms by *in vitro* and *in vivo* studies. EUE and its two active constituents, aucubin and geniposide, inhibited palmitate-induced endoplasmic reticulum (ER) stress, reducing hepatic lipid accumulation through secretion of apolipoprotein B and associated triglycerides and cholesterol in human HepG2 hepatocytes. To determine how EUE diminishes the ER stress response, lysosomal and proteasomal protein degradation activities were analyzed. Although proteasomal activity was not affected, lysosomal enzyme activities including V-ATPase were significantly increased by EUE as well as aucubin and geniposide in HepG2 cells. Treatment with the V-ATPase inhibitor, bafilomycin, reversed the inhibition of ER stress, secretion of apolipoprotein B, and hepatic lipid accumulation induced by EUE or its component, aucubin or geniposide. In addition, EUE was determined to regulate hepatic dyslipidemia by enhancing lysosomal activity and to regulate ER stress in rats fed a high-fat diet. Together, these results suggest that EUE and its active components enhance lysosomal activity, resulting in decreased ER stress and hepatic dyslipidemia.

## Introduction

Nonalcoholic fatty liver disease (NAFLD) is one of the most common chronic liver disorders [1]. NAFLD is clearly associated with features of Metabolic Syndrome including obesity, type 2 diabetes, hypertension, and dyslipidemia. Hepatic steatosis is considered to be the first stage of NAFLD and often leads to more severe complications including steatohepatitis, cirrhosis, and hepatocellular carcinoma [2]–[4]. Thus, a growing number of studies looking at the mechanism of hepatic steatosis are focused on the causative role of ER stress.

When the ER receives extracellular stress signals, the unfolded protein response (UPR) relieves stress from protein misfolding in the ER. Specifically, the expression of protein kinase-like ER kinase (PERK) and the phosphorylation of eukaryotic initiation factor 2α (p-eIF2α) are increased during chronic ER stress, attenuating new protein synthesis [5]. The UPR regulates genes involved in the transport of unfolded proteins out of the ER as well as in the degradation of these unfolded proteins by ER-associated degradation (ERAD) [6]. The ERAD I is a proteasome/ubiquitination pathway, while the ERAD II pathway is a lysosomal activity pathway [7]. The ERAD mechanism increases the protein folding capacity by reducing protein folding loads [7], [8], implying that ERAD is a physiological pathway that can regulate ER stress responses [8], [9]. Events that disturb ER protein folding and induce the UPR include an altered redox state, calcium equilibrium, and protein degradation. Likewise, accumulation of fatty acids or triglycerides is related to alteration of secretory apo-lipoproteins such as ApoB, which can also induce the UPR and cause hepatic steatosis.

The secretion of ApoB-containing lipoproteins involves co- and post-translational processes. Unassembled or aberrantly expressed ApoB retained in the ER is typically degraded, and, under mild physiological stress, the degradation process is highly activated as an adaptive response that involves both ER resident molecular chaperones such as calnexin and calreticulin as well as ER proteases such as ER 60 [10], [11]. However, under pathological ER stress conditions not regulated by the adaptive response, the physiological degradation machinery does not function efficiently, leading to accumulation of unfolded proteins including ApoB [12]. During this type of ER stress, hepatic lipid synthesis and secretion may also be affected by the alteration of secretory ApoB protein folding processes [13]. Therefore, it is necessary to study ER stresses to determine how to control pathological ER stress phenomena such as hepatic steatosis.

*Eucommia* cortex obtained from the bark of 15–20-year-old *E. ulmoides* Oliver trees [14] is a traditional medicine used in Korea, Japan, and China. According to ancient records, roasted *Eucommia* cortex is recommended for reinforcing muscles and lungs, lowering blood pressure, preventing miscarriages, improving the tone of the liver and kidneys, and increasing longevity [15]. Du-zhong (*E. ulmoides* Oliver) leaves containing many of the same components as the *Eucommiae* cortex have recently become a focus of medical research [16]. Indeed, *E. ulmoides* Oliver tea, an aqueous extract of *E. ulmoides* Oliver leaves, is known as a functional health food and is commonly used for the treatment of hypertension [17]. Likewise, extracts of *E. ulmoides* Oliver leaves have been suggested to have recuperative effects for hypercholesterolemia and fatty liver disease [18]. *E. ulmoides* Oliver contains many phytochemicals such as polyphenolics, flavonoids, and triterpenes [19]. Flavonol glycosides from *E. ulmoides* Oliver have been reported to inhibit glycation and to prevent diabetes [20], [21]. Yen and Hsieh [14] reported that water extracts of *E. ulmoides* Oliver leaves have antioxidant activity toward various lipid peroxidation models, with a good correlation between the polyphenol content of water extracts and observed antioxidant activity.

Based upon these observations, we examined the potential regulatory effects of *E. ulmoides* Oliver on hepatic dyslipidemia. We found that *E. ulmoides* Oliver significantly regulated hepatic lipid accumulation both *in vitro* and *in vivo*. Our study results suggest that the regulatory mechanism of *E. ulmoides* Oliver and its active constituents, aucubin and geniposide [22], [23], toward hepatic dyslipidemia involves regulation of ER stress and associated lysosomal activity.

## Materials and Methods

### Materials

*E. ulmoides* Oliver extracts (EUE) were obtained from the Korea Research Institute of Bioscience & Biotechnology (Daejeon, Korea). Extracts were prepared by ethanol extraction of *E. ulmoides* Oliver extracts (200 g) by sonicating with 100% methanol (1g: 8 mL) for 3 days. After filtration, the solvent phase of the filtrate was concentrated by freeze-drying, and the final EUE was obtained and stored at −4°C. For animal experiments, powdered EUE was weighed and re-extracted with 25% ethanol for 2 hours at 90°C using a reflux apparatus. The extract was then filtered, evaporated under vacuum, pulverized, and stored at 4°C. Bafilomycin, aucubin, and geniposide were obtained from Sigma Chemical Company (St. Louis, MO). Antibodies against the 20S core proteasome subunit and carbobenzoxy-Leu-Leu-Glu-7-amino-4-methylcoumarin (Z-LLE-AMC) were from Enzo Life Sciences (Farmingdale, NY). LysoTracker Red DND-26 was from Molecular Probes (Eugene, OR). Kits for measuring total levels of cholesterol and triglyceride were from Asan Pharmaceutical Company (Seoul, Korea). Phosphate-buffered saline (PBS) was purchased from Invitrogen (Carlsbad, CA). Poly-(I:C) and trypan blue dye were from Sigma-Aldrich (St. Louis, MO). All other chemicals were of analytical grade and were purchased from Sigma.

### Cells

Human hepatocellular carcinoma cells (HepG2) were cultured in Dulbecco's modified Eagle Medium (DMEM) (Invitrogen) with 10% fetal bovine serum (FBS) (Biomeda Corp, Foster City, CA) and penicillin-streptomycin (penicillin: 10,000 U/mL, streptomycin: 10,000 μg/mL) (Invitrogen). Freshly trypsinized HepG2 cells were suspended at 5×10^5^ cells/mL in standard HepG2 culture medium and seeded at 10^6^ cells per well in standard six-well tissue culture plates. Cells were incubated at 37°C in a 90% air/10% CO_2_ atmosphere, and 2 mL of medium was exchanged every other day. HepG2 cells were cultured in standard medium for 2–3 days to 90% confluency before being treated with free fatty acids and other additives. HepG2 cell viability was determined by trypan blue dye exclusion using a hemocytometer.

### Animal Treatment and Care

Female Sprague-Dawley rats weighing 250–270 g were obtained from Damul Science Co (Daejeon, Korea). Rats were maintained on a 12∶12-hours light:dark cycle (lights on at 06∶00) in stainless steel wire-bottomed cages and acclimated under laboratory conditions for at least 1 week before experiments. Rats were fed an appropriate diet with free access to water and were weighed weekly. All animal procedures for this study were performed in accordance with the regulations of the care and use of laboratory animals guide of Chonbuk National University and were approved by the Chonbuk National University laboratory animal center of the Institutional Animal Care and Use Committee (IACUC, CBU 2013–0015), and all efforts were made to minimize animal suffering. The control group (n = 10) was fed a standard diet, while the high-fat diet (HFD) group (n = 12) was fed a calorie-rich diet composed of 1% cholesterol, 18% lipid (lard), 40% sucrose, 1% AIN-93G vitamins, and 19% casein. The fiber and mineral contents were the same in both the control and high-fat diets. Rats in the EUE-25 group (n = 10) and control group (n = 10) were fed an HFD with 0.25, 0.5, or 1 g/kg EUE-25. Experiments were terminated after 10 weeks, and serum samples were collected and measured for cholesterol, triglyceride, and liver lipid contents. In addition, tissues were homogenized for Western blot analysis.

### Animal Sacrifice

Rats were anaesthetized with diethyl ether (Sigma) and sacrificed by cervical dislocation. Tissues and blood samples were collected from all sacrificed animals. Whole blood was immediately placed on ice in a 1.5 mL centrifuge tube for 15 to 30 min and spun at 8,000 rpm for 10 min. Sera were then transferred to fresh 1.5 mL centrifuge tubes and stored at −80°C. All harvested tissues were immediately placed in liquid nitrogen and stored at −80°C.

### Histological Analysis

Liver samples were fixed in 10% formalin and embedded in paraffin. Liver sections were incubated for 10 min in 0.5% thiosemicarbazide, stained with 0.1% Sirius red F3B in saturated picric acid for 1 hours, and washed with acetic acid (0.5%). Sections were visualized using a Nikon Eclipse E600 microscope (Kawasaki, Kanagawa, Japan) at 40× magnification, and relative areas of fibrosis (% positive areas for Sirius red staining) were quantified by histomorphometry using a computerized image analysis system (AnalySIS, Soft Imaging System, Munster, Germany). Hepatic steatosis was assessed by Oil Red O staining. Briefly, liver cryosections were fixed for 10 min in 60% isopropanol followed by staining with 0.3% Oil Red O in 60% isopropanol for 30 min and were then washed with 60% isopropanol. Sections were counterstained with Gill's hematoxylin, washed with acetic acid (4%), and mounted with an aqueous solution. Stained sections were quantified by histomorphometry.

### Immunoblotting

HepG2 cells were washed twice with cold PBS and lysed in 300 μL/well CelLytic M cell lysis buffer (Sigma-Aldrich) supplemented with protease inhibitor cocktail (Roche Applied Science, Indianapolis, IN). Cell lysates were clarified by centrifugation at 12,000 rpm for 30 min, and the supernatant was collected. Total protein was quantified using a BCA assay kit (Pierce Inc., Rockford, IL). Lysates (45 μg) were resolved by SDS-PAGE (Bio-Rad) and then transferred to nitrocellulose membranes. Membranes were blocked for 1 hours with 5% skim milk in Tris-buffered saline (0.137 M NaCl, 0.025 M Tris, pH 7.4) containing 0.1% Tween-20 (T-TBS). Primary antibodies consisted of mouse anti-amylase, mouse anti-eIF2α, rabbit anti-ATF6α, mouse anti-GADD153/C/EBP homologous protein (CHOP), mouse anti-GRP78, β-actin (Santa Cruz Biotechnologies, Inc., Santa Cruz, CA), and rabbit anti-phospho-eIF2 and rabbit anti-IRE1α (Cell Signaling. Technologies, Inc., Danvers, MA). Antibodies were diluted according to the manufacturers' recommended protocols. Protein signals were visualized using enhanced chemiluminescence (ECL) reagent (SuperDetect^TM^ ECL Western Blotting Detection Reagent, DaeMyung Science Co., Ltd, Seoul, Korea). Finally, membranes were exposed to imaging film (Kodak BioFlexEcono Scientific Supplies, Citrus Heights, CA) and developed using a Kodak X-OMAT 1000A Processor.

### Oil Red O Staining

To measure cellular neutral lipid droplet accumulation, HepG2 cells were stained using Oil Red O. After treatment, cells were washed three times with ice cold PBS and fixed with 10% formalin for 60 min. After fixation, cells were washed and stained with Oil Red O solution (stock solution, 3 mg/mL in isopropanol; working solution, 60% Oil Red O stock solution and 40% distilled water) for 60 min at room temperature. After staining, cells were washed with water to remove unbound dye. To quantitate Oil Red O content levels, isopropanol was added to each sample, and samples were shaken at room temperature for 5 min. Oil Red O levels were determined by spectrophotometry at 510 nm.

### Measurement of Total Lipid, Triglyceride, and Cholesterol Levels

For lipid determination, cell or rat liver homogenates were extracted according to a modified Bligh and Dyer procedure [24]. Samples were homogenized with chloroform-methanol-water (8∶4∶3), shaken at 37°C for 1 hours, and centrifuged at 1,100×*g* for 10 min. The bottom layer was collected and suspended for hepatic lipid analysis. Triacylglycerol, total cholesterol, and total lipid contents were measured using kits from Randox Laboratories (Antrim, UK) in accordance with the manufacturer's instructions.

### Lysosomal Isolation

Lysosomal isolation was performed according to a published protocol [12]. Briefly, cells were rinsed in cold STE buffer (0.25 M sucrose, 0.01 M Tris-HCl, 1 mM EDTA, and 0.1% ethanol) and scraped into a dish containing 1 mL STE buffer and protease inhibitors (Sigma-Aldrich). The cell suspension was disrupted in a Kontes cell disruption chamber using three 20 min passes at 150 psi. This method consistently disrupted >95% of cells while leaving the lysosomes intact. The resulting suspension was centrifuged at 1000×*g* to separate post-nuclear supernatant and nuclear pellet. Post-nuclear supernatant density was increased to 1.15 g/mL with sucrose and applied to a sucrose density gradient from 1.28 to 1.00 μg/mL, which was then centrifuged at 64,000×*g* for 4 hours at 4°C to isolate the lysosomal fraction.

### Microscopic Assessment of Lysosome Activity

A time course of lysosomal activity was determined by staining with LysoTracker Red (577/590 nm). Cells were grown in cell culture dishes, rinsed with PBS, and stained with 100 nM LysoTracker Red DND-26 (Molecular Probes, Eugene, OR) in serum-free medium for 30 min at room temperature, followed by washing with PBS. Red fluorescent images were acquired using a digital CCD color video camera CCS-212 (Samsung, Seoul, Korea) and transferred to a computer with a WinFast 3D S680 frame grabber (Leadtek, Taipei, Taiwan). Fluorescence values of 100 randomly selected cell images were measured for each treatment condition. Lysosome fluorescence intensity was expressed as a ratio of the average fluorescence of 100 treated cells to the fluorescence of 100 control cells. Localization of cathepsin B and LAMP-1 was determined by immunofluorescence confocal microscopy. Cells were cultured and fixed with methanol for 10 min at room temperature. After permeabilization with Triton X-100 (0.1%), cells were incubated with PBS containing 3% BSA for 30 min at room temperature. Cells were then double-stained for 2 hours at room temperature in PBS-3% BSA with primary antibodies: anti-LAMP-1 rabbit (1∶100, Millipore, MA) or anti-cathepsin B (15 μg/mL, R&D Systems, MN). Immunofluorescence staining was performed with secondary antibodies in PBS-0.5% BSA for 60 min at room temperature. Slides were mounted with Aqua Poly/Mount (Polysciences), and images were acquired using a Delta Vision Spectris Image Deconvolution System on an Olympus IX70 microscope with Softworx Explorer software from Applied Precision.

### Lysosomal Enzyme Activity Assays

Lysosomal enzyme assays were performed at 35°C with p-nitrophenyl-derivatized monosaccharide substrates, as previously described [25]. Enzymatic reactions were terminated by the addition of an equal volume of 1 M Na_2_CO_3_. Released p-nitrophenol was measured by spectrophotometry at 420 nm, with activity units defined as nanomoles of p-nitrophenol released per min.

### Statistical Analysis

Results are presented as the mean ± SEM. MicroCal Origin software (Northampton, MA) was used for statistical calculations. Differences were tested for significance using one-way analysis of variance (ANOVA) with Duncan's multiple range test. Statistical significance was set at *p*<0.05.

## Results

### EUE inhibits palmitate-induced ER stress response

*E*. Oliver extracts (EUE) are known to have anti-hyperlipidemic properties; however, the mechanisms by which EUE mediates these effects are unknown [18]. In this study, EUE was applied to a model of palmitate-induced ER stress and its associated lipid accumulation. To confirm that non-toxic concentrations and time periods were chosen for palmitate treatment, HepG2 cells were exposed to palmitate at 300 or 500 μM for 0, 12, 24, 36, or 48 hours. Treatment with 300 μM palmitate for 12 hours was selected as the optimal nontoxic condition for studying lipid metabolism (Figure S1). Among the ER stress responses, phosphorylation of PERK and eIF2α was markedly increased in cells treated with 300 μM palmitate. Pretreatment with EUE inhibited phosphorylation of PERK and expression of its downstream effectors, eIF2α and CHOP (Figs. 1 A and B). However, other ER stress signaling proteins, namely ATF6, IRE-1α, and GRP78, were not affected by treatment with palmitate.

**Figure 1:** *E. ulmoides* Oliver extracts inhibit palmitate-induced ER stress response. (A) Cells were treated with 300 μM palmitate and 0, 25, 50, or 100 μg/mL extract for 12 hours. Immunoblotting was performed using antibodies against GRP78, PERK, p-PERK, CHOP, IRE1α, p-eIF2α, eIF2α, or β-actin. (B) Cells were treated with 300 μM palmitate in the presence of 100 μg/mL EUE for 0, 3, 6, 9, 12, 18, or 24 hours. Quantification of immunoblot data is shown (right panel). Immunoblotting was performed with antibodies against GRP78, PERK, p-PERK, CHOP, IRE1α, p-eIF2α, eIF2α, or β-actin. Data shown are the mean ± SE of three independent experiments, each performed with triplicate biological replicates. ^*^ *p*<0.05, significantly different from cells treated with palmitate alone at the corresponding time point. Pal, palmitate; EUE, *E. ulmoides* Oliver extract.

### EUE regulates lipid metabolism

To investigate the ability of EUE to regulate lipid accumulation, HepG2 cells were treated with palmitate to induce hepatic lipid accumulation. Treatment of HepG2 cells with EUE and a nontoxic concentration of palmitate (300 µM) significantly inhibited palmitate-induced cellular lipid accumulation (Fig. 2A). To investigate the mechanism of this inhibition, apolipoprotein pathways were examined because dysregulation of apolipoprotein secretion is related to ER stress and hepatic accumulation [26]. Expression of ApoA1 and ApoB was analyzed after treatment with 100 μg/mL EUE with or without palmitate. Expression of ApoB but not ApoA1 was increased in cell lysates after palmitate treatment (Fig. 2B). Likewise, treatment with EUE regulated the change in ApoB expression. Specifically, the level of secreted ApoB in the medium was decreased in the presence of palmitate without EUE but increased in a time-dependent manner after treatment with EUE. Levels of triglycerides and cholesterol were measured for cell lysates and media from palmitate-treated cells with or without EUE treatment. The levels of intracellular triglyceride and cholesterol were strongly increased in palmitate-treated cells, whereas this increase was prevented by EUE (Fig. 2C). In media samples, triglyceride and cholesterol levels were significantly decreased by treatment with palmitate and, consistent with our ApoB expression results, were recovered by treatment with EUE.

**Figure 2:** *E. ulmoides* Oliver extract reduces hepatic lipid accumulation and levels of secreted apolipoprotein B. (A) Cells were treated with 300 μM palmitate in the absence or presence of 100 μg/mL EUE for 12 hours. Fat accumulation was determined by Oil Red O staining. Images of cells were obtained at 200X original magnification and used for quantitative analysis of cellular lipid deposition (right). ^*^ *p*<0.05, significantly different from cells treated with palmitate alone. (B) Cells were treated with 300 μM palmitate in the presence or absence of 100 μg/mL EUE for 0, 3, 6, 9, 12, 18, or 24 hours. Cell lysates and media samples were subjected to immunoblot analysis with anti-ApoA1 or anti-ApoB. CBB staining was performed as an equal loading control. (C) Cells were treated with 300 μM palmitate in the absence or presence of 100 μg/mL EUE for 0, 6, 12, 24, or 48 hours. Triglyceride and cholesterol levels were measured for both cell lysates and media alone. ^*^ *p*<0.05, significantly different from cells treated with palmitate alone at the corresponding time point. Pal, palmitate; EUE, *E. ulmoides* Oliver extracts; CBB, Coomassie brilliant blue.

### Aucubin and geniposide from EUE inhibit palmitate-induced phosphorylation of PERK and eIF2α

We next examined the effects of aucubin and geniposide, the major active constituents of EUE, on palmitate-associated lipid metabolism. First, we co-treated cells with palmitate and either aucubin or geniposide. Neither aucubin nor geniposide affected cell viability in the presence of palmitate (Figure S2). We then exposed cells to palmitate in the presence or absence of 10 μg/mL of aucubin or geniposide and examined the ER stress response. Phosphorylation of PERK and eIF2α was markedly increased in cells treated with 300 μM palmitate, while expression of other ER stress signaling proteins, namely ATF6, IRE-1α and GRP78, were not affected. Conversely, co-treatment with aucubin or geniposide inhibited phosphorylation and downstream signaling of PERK, eIF2α, and CHOP (Fig. 3).

**Figure 3:** Aucubin and geniposide inhibit palmitate-induced ER stress response. Cells were treated with 300 μM palmitate in the absence or presence of 10 ug/mL aucubin or geniposide for 0, 3, 6, 9, 12, 18, or 24 hours. Immunoblotting was performed using antibodies against GRP78, PERK, p-PERK, CHOP, IRE1α, p-eIF2α, eIF2α, or β-actin. Quantification of immunoblot data is shown (lower panel). ^*^ *p*<0.05, significantly different from cells treated with palmitate alone at the corresponding time point. Pal, palmitate; EUE, *E. ulmoides* Oliver extracts.

### Aucubin and geniposide regulate lipid metabolism

We examined the effects of aucubin and geniposide on hepatic lipid accumulation. Treatment with aucubin and geniposide in the presence of 300 μM palmitate significantly inhibited palmitate-induced cellular lipid accumulation as determined by Oil Red O staining (Fig. 4A). Expressions of ApoA1 and ApoB were also analyzed after treatment with aucubin or geniposide in the presence or absence of palmitate. Co-treatment of cells with palmitate and either aucubin or geniposide inhibited palmitate-induced expression of ApoB (Fig. 4B). In culture media, expression of ApoB but not ApoA1 was increased in a time-dependent manner by 10 μg/mL aucubin or geniposide under palmitate-treatment conditions. The levels of triglycerides and cholesterol are shown in Fig. 4C; these levels were strongly increased in 300 μM palmitate-treated cells but were ameliorated by 10 μg/mL aucubin or geniposide. Consistent with the ApoB expression results, levels of triglycerides and cholesterol in media were significantly decreased by palmitate, whereas treatment with aucubin or geniposide prevented this decrease (Fig. 4B).

**Figure 4:** Aucubin and geniposide reduce hepatic lipid accumulation and secretion of apolipoprotein B. (A) Cells were treated with 300 μM palmitate in the absence or presence of 10 μg/mL aucubin or geniposide for 12 hours. Fat accumulation was determined by Oil Red O staining. Images of cells were obtained at 200X original magnification and used for quantitative analysis of cellular lipid deposition (lower panel). ^*^ *p*<0.05, significantly different from cells treated with palmitate alone. (B) Cells were treated with 300 μM palmitate in the presence or absence of 10 μg/mL aucubin or geniposide for 0, 3, 6, 9, 12, 18, or 24 hours. Cell lysates and medium were immunoblotted with anti-ApoA1 or anti-ApoB, and CBB staining was performed separately as an equal loading control. (C) Cells were treated with 300 μM palmitate in the presence or absence of 10 μg/mL aucubin or geniposide for 0, 6, 12, 24, or 48 hours. Triglycerides and cholesterol were measured in cell lysates and media alone. ^*^ *p*<0.05, significantly different from cells treated with palmitate alone at each corresponding time point. Pal, palmitate; CBB, Coomassie brilliant blue.

### EUE, aucubin, and geniposide enhance lysosomal activity

We were interested in how EUE regulates ER stress (Fig. 1B). Because enhanced protein degradation has been demonstrated to relieve ER stress [27], we investigated proteasomal and lysosomal degradation. In palmitate-treated cells, proteasomal activity was not affected by EUE, aucubin, or geniposide (Figure S3). We then used lysoTracker dye to evaluate lysosomal activity in HepG2 cells, which decreased significantly after treatment with palmitate (Fig. 5A). Treatment with EUE, aucubin, or geniposide clearly reversed the decrease in fluorescence in palmitate-treated cells (Fig. 5B).

**Figure 5:** *E. ulmoides* Oliver extract, aucubin, and geniposide enhance lysosomal activity. (A) Cells were treated with 100 μg/mL EUE, 10 μg/mL aucubin, or 10 µg/mL geniposide in the presence or absence of 300 µM palmitate for 12 hours, followed by exposure to 5 μM LysoTracker and image acquisition and quantification (lower panel). (B) Cells were fixed and immunostained with antibodies for cathepsin B or Lamp-1. Quantification of fluorescence is shown (lower). (C) The activities of α-mannosidase, β-galactosidase, and β-glucuronidase were analyzed from lysosomal extracts of cells treated for the indicated time periods. ^*^ *p*<0.05, significantly different from cells treated with palmitate alone (A, B); ^*^ *p*<0.05, significantly different from cells treated with palmitate alone at each corresponding time point (C). DIC, differential interference contrast microscopy; Pal, palmitate; EUE, *E. ulmoides* Oliver extract.

To evaluate the effect of EUE on lysosomal degradation, we used the representative lysosomal enzyme Cathepsin B [28]. Immunostaining analysis with antibodies to cathepsin B and lysosomal-associated membrane protein 1 (Lamp-1), a lysosomal marker, revealed decreased fluorescence of cathepsin B in palmitate-treated cells (Fig. 5B). The decreased fluorescence of cathepsin B was reversed by co-treatment with EUE and aucubin or geniposide. Colocalization of cathepsin B with Lamp-1 was observed in all treatment groups, suggesting that palmitate affected lysosome function but did not influence lysosomal membrane permeability. To confirm these results, we evaluated several other lysosomal enzymes, namely, β-galactosidase, α-mannosidase, and β-glucuronidase. These enzymes were inhibited by palmitate treatment in a time-dependent manner (Fig. 5C). However, in cells exposed to EUE, aucubin, or geniposide in the presence of palmitate, the activities of α-mannosidase, β-glucuronidase, and β-glucuronidase were relatively stable compared to levels observed after treatment with palmitate alone.

### The lysosome inhibitor bafilomycin reverses the effects of EUE on the ER stress response and lipid metabolism

V-ATPase maintains the acidic pH of the lysosome and is a representative lysosomal protein [29]. To understand the role of lysosomes in ER stress-associated dyslipidemia, we used the V-ATPase inhibitor bafilomycin. Specifically, we evaluated the effect of bafilomycin on the ER stress response in palmitate-exposed HepG2 cells. Treatment of cells with bafilomycin and EUE significantly reversed the effect of EUE against the ER stress response as determined by measuring the expression of p-PERK, p-eIF-2α, and CHOP (Fig. 6A). Likewise, bafilomycin markedly reversed EUE-induced cellular lipid accumulation, as shown by Oil Red O staining (Fig. 6B). Bafilomycin also reversed EUE-induced intracellular ApoB accumulation (Fig. 6C). Treatment with 10 nM bafilomycin decreased the levels of secreted ApoB but not ApoA1 in the media of cells co-treated with EUE and palmitate (Fig. 6C, lower). We consistently observed increased accumulation of intracellular triglyceride and cholesterol with bafilomycin treatment in cells co-treated with EUE and palmitate compared to cells not treated with bafilomycin (Fig. 6D, left). The levels of triglycerides and cholesterol secreted into the culture media decreased significantly after treatment with bafilomycin, confirming that the lipid secretion pathways were dysregulated by the lysosomal V-ATPase inhibitor (Fig. 6D, right). The V-ATPase inhibitor, bafilomycin, similarly reversed the component of EUE, aucubin or geniposide-induced regulation against lipid accumulation processes in palmitate-treated cells. Together, these data suggest that enhanced V-ATPase activity is necessary for EUE to diminish the ER stress response and associated hepatic lipid accumulation.

**Figure 6:** Bafilomycin reverses *E. ulmoides* Oliver extract-induced regulation of ER stress and lipid accumulation. (A) Cells were treated with 300 μM palmitate and 100 μg/mL EUE, 10 μg/mL aucubin, or 10 μg/mL geniposide in the presence or absence of 10 nM bafilomycin for 12 hours. Immunoblotting was performed using antibodies against GRP78, PERK, p-PERK, CHOP, IRE1-α, p-eIF2α, eIF2α, or β-actin. (B) Images were obtained at 200X magnification for determination of fat accumulation by Oil Red O staining. (C) Cell lysates and media were immunoblotted with anti-ApoA1 or anti-ApoB. (D) Triglycerides and cholesterol levels in lysates or media were measured as described in the Materials and Methods. ^*^ *p*<0.05, significantly different from cells treated with palmitate alone. Values are the mean±SE of three independent experiments. Con, control; Pal, palmitate; EUE, *E. ulmoides* Oliver extracts; Au, aucubin; Geni, geniposide; Bafi, Bafilomycin; CBB, Coomassie brilliant blue staining.

### EUE reduces hepatic lipid accumulation and stimulates lysosome activity in high-fat-diet-fed rats

To examine the physiological relevance of our *in vitro* observations, we examined the effect of EUE on hepatic dyslipidemia in high-fat-diet (HFD)-fed rats. For *in vitro* experiments, *E. ulmoides* cortex was re-extracted with various ethanol/water mixtures (25, 50, 75, or 100% ethanol v/v) by reflux. The aucubin and geniposide contents in the extracts were measured by HPLC to determine the amount of extract to use for animal experiments. We found no significant difference in the content of geniposide extracted (Figure S4) according to the amount of ethanol. Conversely, we measured the highest content of aucubin in the 25% ethanol extract, suggesting a positive correlation with triglycerides and total cholesterol secretion activity, especially for the 25% ethanol extract in palmitate-treated hepatic cells (Figure S5). Based on these results, the EUE with the highest abundance of active compound was orally administered (0.25, 0.5 and 1 g/kg/day) to HFD rats. Body weight was reduced in EUE-treated HFD rats compared to HFD-only controls (Figure S6). The liver weights exhibited tended to be less in EUE-treated HFD rats compared to HFD-only controls (Figure S6). We next examined whether EUE affects the HFD-induced ER stress response *in vivo*. The ER stress response was diminished by EUE as determined by expression of p-PERK, p-eIF2α, and CHOP (Fig. 7A). Lysosomal activity was also analyzed *in vivo* to identify a possible mechanism for regulation of ER stress by EUE. Consistent with our *in vitro* data, the activities of the lysosomal enzymes α-mannosidase, β-glucuronidase, and β-galactosidase were reduced in HFD rats and were restored by treatment with EUE (Fig. 7B). Analysis of hepatic lipid accumulation was also determined. Oil Red O staining indicated that hepatic lipid accumulation was reduced in EUE-treated HFD rats (Fig. 7C). Consistent with these results, EUE markedly decreased hepatic lipid content as determined by hepatic triglyceride and cholesterol levels (Fig. 7D). Conversely, EUE increased total plasma triglyceride and cholesterol levels. Expression of hepatic ApoB, the lipoprotein for LDL and triglycerides, was increased in HFD-fed rats, while levels of ApoA1 were unaffected (Fig. 7E). Further, in plasma, ApoB expression was decreased in HFD-fed rats, while the level of ApoA1 was not affected. Lastly, treatment with EUE reversed the dysregulated secretion of ApoB in both the liver and serum.

**Figure 7:** *E. ulmoides* Oliver extract regulates ER stress and hepatic lipid accumulation and enhances lysosome activity in high-fat-diet rats. Rats were fed a normal or high-fat diet with 0, 0.25, 0.5, or 1 g/kg EUE for 10 weeks, after which livers were isolated. (A) Immunoblotting was performed with antibodies against GRP78, PERK, p-PERK, CHOP, IRE1-α, p-eIF2α, eIF2α, or β-actin. (B) Lysosome fractionation was performed using liver samples, and the activities of α-mannosidase, β-glucuronidase, and β-galactosidase were subsequently determined. (C) Livers were stained with Oil Red O dye, and images were obtained at 200X magnification to observed hepatic fat accumulation. (D) Triglyceride and cholesterol levels were measured in both the liver and plasma. (E) Immunoblotting was performed with ApoA1 or ApoB antibodies using liver and plasma samples. ^*^ *p*<0.05, significantly different from the control group at each corresponding time point. CV, central vein; Con, control; HFD, high-fat-diet; EUE, *E. ulmoides* Oliver extract.

## Discussion

In this study, we examined the effects of EUE on hepatic dyslipidemia both *in vitro* and *in vivo*. EUE diminished the palmitate-induced ER stress response, expression of associated lipogenic genes, and apolipoprotein secretion through enhancement of lysosomal V-ATPase activity. Consistent with these observations, aucubin and geniposide influenced fatty acid-induced ER stress and hepatic dyslipidemia through a similar mechanism, namely, lysosome activation and suppression of ER stress.

The expression of p-eIF2α and CHOP increased in cells exposed to palmitate (Fig. 1B, Fig. 3), suggesting activation of a PERK-dependent pathway among the ER stress response signal transductions. Although significant activation of additional ER stress pathways has been observed in pancreatic beta-cell system [30], activation of components of the ER stress pathway by palmitate has previously been thought to be primarily confined to a PERK-dependent process [31]–[33]. Indeed, the specific PERK-eIF2α-CHOP ER stress arm was stimulated without affecting expression of GRP78, IRE-1α, or ATF6. More specifically, PERK siRNA has been shown to abrogate lipid accumulation [31]. The application of a nontoxic concentration of palmitate in our experiments (Figure S1) may explain the specific PERK-ER stress arm activation. The PERK-eIF2α-CHOP axis may be the primary mechanistic target of EUE against hepatic dyslipidemia.

EUE regulates the ER stress response, alters apolipoprotein secretion, and influences hepatic lipid accumulation in palmitate-treated cells (Fig. 2A). ER stress-associated alteration of ApoB secretion may explain the relationship between ER stress and hepatic steatosis. In our study, we utilized the specific conditions of palmitate-associated ER stress altering ApoB secretion, which, in turn, lead to hepatic lipid accumulation. The alteration of apolipoprotein secretion and subsequent lipid accumulation were inhibited by EUE (Figs. 2B, 2C). It has been suggested that ER stress-associated hepatic lipid accumulation is related to a reduction of ApoB secretion [26]. Accumulating evidence suggests an association between ER stress and secretory protein alterations [12]. Thus, EUE-induced ER stress regulation may also contribute to reduction of lipid accumulation through alteration of apolipoprotein secretion.

Our observations of lysosomal activity may explain how EUE regulates the ER stress response and dysregulation of ApoB. Lysosomal activity was significantly decreased upon exposure to palmitate; however, in the presence of EUE, lysosomal activity was only slightly affected by exposure to free fatty acids (Fig. 5C). Thus, the role of EUE on reestablishing ER homeostasis by enhancing lysosomal activity may lead to the amelioration of ER stress and subsequently alleviate hepatic dysfunction, e.g., lipid accumulation.

Lysosome-associated protein degradation also functions as a cytoplasmic quality control mechanism to eliminate protein aggregates and damaged organelles [28], [29]. Although non-lysosomal functions are required for the degradation of short-lived proteins in the cytosol as well as for the stress-induced enhancement of degradation of cellular proteins within lysosomes [34], lysosomal functions appear to reflect a reduced ER stress response under EUE-treated conditions. Throughout this study, we observed high lysosomal activity that explained how EUE regulates the ER stress response. Basally increased lysosomal function is a key phenomenon of the EUE single-treatment condition (Figs. 5A, B). When exposed to free fatty acids, EUE may reduce the folding load of altered/damaged proteins through the highly activated ERAD II pathway, leading to the amelioration of ER stress and hepatic lipid accumulation. Defects in the ERAD II system enhance the ER stress response, leading to dyslipidemia [30]. ER stress itself has been correlated with hepatic steatosis, but the basic mechanism regarding induced ER stress response has not been elucidated. Puri and colleagues [35] recently examined a potential role of ER stress in human NAFLD and found that the degree of UPR activation in liver biopsies from patients with NAFLD is variable compared to those from subjects with metabolic syndrome or normal liver histology. Further, they determined that human NASH was specifically associated with the activation of C-jun N-terminal kinase (JNK), an ER stress-associated stress protein. However, any induction mechanism or regulatory pathway of the ER stress in hepatic dyslipidemia has not been determined. An alteration of ERAD II activity needs to be considered as a possible mechanism for hepatic ER stress, as strategies capable of maintaining lysosomal activity appear to be necessary for successful treatment of hepatic lipid accumulation.

The effects of EUE were also investigated in an HFD-induced ER stress and liver steatosis model *in vivo*. Our *in vitro* results clearly showed that the geniposide and aucubin components of EUE contributed significantly to amelioration of intracellular lipid accumulation, and thus an ethanol extract of EUE with the highest content of active the compound aucubin was selected for animal experiments. An HFD can be used to experimentally induce liver steatosis in an acute setting [36], [37]. Lysosome activity was transiently decreased after administration of an HFD (Fig. 7B). However, EUE dose-dependently enhanced the activity of lysosomal enzymes, including α-mannosidase, β-glucuronidase, and β-galactosidase, in HFD rats, linking it to suppression of ER stress, induction of associated lipogenic genes, alteration of protein secretory pathways, and hepatic lipidemia.

In conclusion, the results of our study show that EUE inhibits liver steatosis. Further, our results suggest that EUE and its active components, aucubin and geniposide, are ER stress suppressors. The mechanism of ER stress suppression by EUE and its active compounds was associated with enhancement of lysosomal activity, including that of V-ATPase. Through more efficient protein degradation resulting from treatment with EUE, aucubin, or geniposide, demands on ER protein folding might be lessened, leading to a relieved ER stress response. Our findings provide molecular evidence for the use of EUE as a possible therapy for the management of hepatic dyslipidemia.

## Supporting Information

Figure S1 ***E. ulmoides*** **Oliver extract protects cells against palmitate.** (A) HepG2 cells were exposed to the indicated concentrations of EUE and cell viability was determined. (B) Cells were exposed to 300 μM or 500 μM palmitate for 0, 12, 24, 36 or 48 hrs and cell viability was determined by trypan blue dye exclusion staining. (C) Cells were exposed to the indicated concentrations of EUE in the presence or absence of 300 μM palmitate. For the control group, cells were treated with vehicle. After 12 h, cell viability was determined by trypan blue dye exclusion staining. ^*^ *p*<0.05, significantly different from non-treated control cells. Pal, palmitate; EUE, *E. ulmoides* Oliver extracts.
(TIF)

Figure S2 **Aucubin and geniposide protects cells against palmitate.** Cells were exposed to 300 μM palmitate and 10 ug/mL of either aucubin or geniposide. Cell viability was determined by trypan blue dye exclusion staining analysis. Pal, palmitate.
(TIF)

Figure S3 ***E. ulmoides*** **Oliver extract, aucubin, and geniposide do not affect proteasome expression or activity.** (A) Proteasomal protein expression was measured by immunoblotting using an antibody against the 20 S core proteasome. (B) Proteasomal activity was determined by fluorescence. Values are the mean ± SE of three independent experiments. Con, control; Pal, palmitate; EUE, *E. ulmoides* Oliver extracts.
(TIF)

Figure S4 **A 25% ethanol extract of** ***E. ulmoides*** **Oliver contains a high amount of Aucubin.** (A) LC spectrum of an aucubin standard. (B) LC spectrum of EUE showing the presence of aucubin. (C) Concentration of aucubin in EUE as a function of the concentration of ethanol used for extraction.
(TIF)

Figure S5 **A 25% ethanol extract of** ***E. ulmoides*** **Oliver significantly regulates hepatic cellular lipid accumulation and contains the highest concentration of aucubin.** Cells were treated with 300 μM palmitate for 12 hrs in the presence or absence of 100 μg/mL ethanol-extracted *E. ulmoides* Oliver in serial dilutions. Triglyceride (A) and total cholesterol (B) were measured in lysates and media. ^*^ *p*<0.05, significantly different from cells treated with palmitate alone. Con, control; Pal, palmitate; EUE, *E. ulmoides* Oliver extracts; Geni, geniposide.
(TIF)

Figure S6 **A 25% ethanol extract of** ***E. ulmoides*** **Oliver regulates body and liver weight in high-fat-diet-treated rats.** Rats in the EUE group (n = 10) were provided a HFD with 0.25, 0.5, or 1 g/kg EUE for 10 weeks. Body weight was measured each week over the 10 week period (A). Liver weight was measured at the end of the 10 week period (B). ^*^ *p*<0.05, significantly different from the control group at each time point (A). ^*^ *p*<0.05, significantly different from control rats (B). Con, control; HFD, high-fat-diet; EUE, *E. ulmoides* Oliver extract.
(TIF)

Methods S1 **Quantitation of aucubin using HPLC-DAD.**
(DOCX)
